This article has been retracted.

# MicroRNA-124 modulates neuroinflammation in acute methanol poisoning rats via targeting Krüppel-like factor-6

**DOI:** 10.1080/21655979.2022.2078549

**Published:** 2022-06-05

**Authors:** Shu Zhou, Jinjun Li, XiaoNa Zhang, Wen Xiong

**Affiliations:** a Department of Emergency, Liuyang People’s Hospita, Liuyang City, Hunan Province, China; b Department of Infectious Diseases, Liuyang People’s Hospita, Liuyang City, Hunan Province, China

**Keywords:** Neuroinflammation, MicroRNA-124, Krüppel-like factor-6, acute methanol poisoning

## Abstract

Microglia activation-stimulated neuroinflammation exerts functionally in neurodegenerative diseases like brain injury. Acute methanol poisoning (AMP) is a crucial cause of death and morbidity that possibly leads to neuroinflammation. Studies have manifested that miRNAs can modulate microglia activation to mediate neuroinflammation. Nevertheless, the role of miR-124 in AMP-stimulated neuroinflammation is uncertain. This research was to explore the action of miR-124 in AMP-stimulated neuroinflammation and its molecular mechanism. The study findings indicated that AMP accelerated microglia activation and stimulated inflammation and oxidative stress in brain tissue of rats. MiR-124 expression was lowered in AMP rats, while KLF6 expression was elevated. Elevated miR-124 or repressed KLF6 increased the number of CD206^+^ cells and decreased the number of CD68^+^ cells, as well as restrained inflammation and NF-κB phosphorylation and induced superoxide dismutase, Nrf2/HO-1, and M2 polarization. MiR-124 modulated microglia activation via targeting KLF6. AMP repressed neuronal viability and enhanced neuronal apoptosis. Suppression of miR-124 further promoted AMP-induced damage to neurons, while inhibition of KLF6 turned around this phenomenon. Anyway, our study demonstrated that miR-124 accelerates M2 polarization via targeting KLF6 to ameliorate AMP-stimulated neuronal damage.

## Highlights

- AMP promotes microglia activation and induces inflammation and oxidative stress.
- AMP induces inhibition of miR-124 expression and promotion of KLF6 expression.
- Overexpression of miR-124 or knockdown of KLF6 promotes microglial M2 polarization and inhibits inflammation and oxidative stress.
- Mir-124 targets KLF6 expression
- miR-124/KLF6 axis affects neuronal viability and apoptosis by regulating microglial polarization.

## 1. Introduction

Methanol is a widely used short-chain fatty alcohol with neurotoxicity. Due to its low cost, it is often used to replace ethanol in industry. However, methanol has great potential safety hazards, and large-scale acute methanol poisoning (AMP) often occurs worldwide [1]. In the liver, the conversion of methanol to formaldehyde by the liver enzyme alcohol dehydrogenase triggers a cascade of metabolic events [2]. As reported, methanol poisoning leads to death, while AMP may result in optic nerve atrophy and cerebral infarction [3]. AMP patients range from dizziness and vomiting to blindness and even death, while survivors also present long-term motor and memory deficits [4]. In addition, AMP causes optic neuropathy and necrosis of the basal ganglia and subcortical white matter [4] and results in an imbalance of oxidative stress in brain tissue, increasing the enrichment of lipid peroxidation products in brain tissue, such as 4-hydroxynonenal and malondialdehyde [5]. It is evident that the accumulation of peroxidation products activates inflammatory signaling pathways in brain tissue, resulting in inflammatory cell infiltration and mediating neuronal apoptosis [6,7].

Microglia are the main innate immune cells in the brain that respond rapidly to pathogens and injury and secrete a variety of pro-inflammatory factors [8]. Microglia acquire different phenotypes including M1 (classical activation) and M2 phenotype (alternative activation) when they receive danger signals [9,10]. The activation of M1 phenotype may be related to inducible nitric oxide synthase and nuclear factor κB (NF-κB) signaling pathways and pro-inflammatory factors like tumor necrosis factor (TNF-α), interleukin (IL-1β), reactive oxygen species (ROS), and nitric oxide synthesis and release [11]. M2 phenotype, defined by alternative and acquired inactivation, promotes phagocytosis of neuronal debris and misfolded proteins, tissue repair, extracellular matrix (ECM) remodeling, anti-inflammatory antagonism of immunosuppression and interaction with IL-10 and transforming growth factor (TGF-β)-associated neuroprotection [12,13]. Microglia activation-stimulated neuroinflammation is the innate immune process protecting the brain from harmful substances [14]. Neuroinflammation is critical in the pathogenesis of neurodegenerative diseases including Parkinson’s disease [15], Alzheimer’s disease [16], and brain injury [17]. Nevertheless, the effect of AMP on microglia and the role of neuroinflammation in AMP-induced brain injury are not yet understood.

MicroRNA (miRNA), a set of short endogenous non-coding RNAs, is available to modulate post-transcriptional genes [18]. Numerous studies have manifested that miRNA is implicated in the process of microglia activation. For instance, neuron-derived exosomes with elevated miR-21-5p accelerate M1 polarization [19], and miR-367 boosts M2 polarization to mitigate inflammatory damage [20]. miR-124 is an essential modulator to mediate microglia activation. Particularly, miR-124 induces M2 polarization to ameliorate cerebral inflammation in cerebral hemorrhage [21]. Nevertheless, the action of miR-124 in AMP-stimulated microglia activation is uncertain.

In this study, the speculation that miR-124 might impact AMP-stimulated neuronal damage by modulating microglia activation was manifested. The influences of miR-124 and its target gene Krüppel-like factor-6 (KLF6) on microglia activation were explored by gain- and loss-of-function experiments. In general, miR-124 accelerated M2 polarization via targeting KLF6, thereby ameliorating AMP-stimulated neuroinflammation.

## 2. Materials and methods

### 2.1. AMP animal model

Male Sprague-Dawley rats (Hunan SJA Laboratory Animal Co., Ltd., Changsha, China) were kept with access to eating and drinking. After 1 week of adaptive feeding (24 ± 2°C, 50–60% humidity, 12-h day–night cycle), the rats were divided into 6 groups (n = 8): control (gavage with equal dose of normal saline with methanol), AMP (gavage with 3 g/kg methanol), miR-124 agomir (injection with miR-124 agomir before gavage with 3 g/kg methanol), agomir negative control (NC) (injection with agomir NC before gavage with 3 g/kg methanol), rAVV-sh-KLF6 (injection with sh-KLF6 recombinant adenovirus vector before gavage with 3 g/kg methanol), and the rAVV-sh-NC (injection with sh-NC recombinant adenovirus vector before gavage with 3 g/kg methanol). After 7-d gavage, the rats were euthanized with excessive CO_2_, and brain tissues were collected, of which one part was fixed with 4% paraformaldehyde for pathological observation and the others were stored for RNA and protein extraction.

### 2.2. Animal treatment

MiR-124 agomir, agomiR NC, rAVV-sh-KLF6, and rAVV-sh-NC were injected into the right ventricle (1.5 mm posterior, 1.5 mm lateral to the bregma, and 2.5 mm deep into the ipsilateral hemisphere). miR-124 agomiR and agomir NC were injected at 1 nmol/d, lasting for 5 d. rAVV-sh-KLF6 and rAVV-sh-NC were injected at 5 × 10^10^ PFU/mL/d, lasting for 2 d.

### 2.3. Immunofluorescence staining

Immunofluorescence staining was implemented as previously described [22]. The brain tissues were cut into 7 μm slices, immersed in 0.1 M phosphate-buffered saline (PBS), and rinsed with 0.2% Triton X-100. After blocking with 5% permeabilized bovine serum albumin, the slices were incubated with the primary antibodies (all Abcam): ionized calcium-binding adapter molecule 1 (Iba-1), CD206 and CD68, as well as the secondary antibody conjugated with Alexa Fluor 488 (#A-21206) and Alexa Fluor 594 (#A-21203) (Invitrogen, USA). Finally, after staining with 4’, 6-diamidino-2-phenylindole (1:300, Cat. #C1002, Beyotime), the images were captured under a fluorescence microscope (Leica DMi8, Leica Microsystems).

### 2.4. Enzyme-linked immunosorbent assay (ELISA)

The brain tissues were homogenized in PBS containing protease inhibitors and centrifuged at 13,000 × g. The supernatant was stored for determining IL-1β, IL-6, TNF-α, malondialdehyde (MDA), and superoxide dismutase (SOD) using ELISA kits (CUSABIO, Wuhan, China) in light of the manufacturer’s instructions [23].

### 2.5. Neuron culture

Neurons PC-12 (American Type Culture Collection, Manassas, VA, USA) were cultured in Dulbecco’s Modified Eagle medium (DMEM) (Gibco) replenished with 10% horse serum and 5% fetal bovine serum (Gibco). The renewal of the medium was performed every 48 h.

### 2.6. Microglial cell culture

Primary microglial cells were isolated from cerebral cortex as previously described [24]. In short, the cerebral cortex was placed in PBS containing 0.25% trypsin, centrifuged, and prepared into a cell suspension at a density of 1 × 10^6^ cells/mL. Subsequently, the cell suspension was mixed with DMEM/F12 (1:1, Gibco). Iba-1, a specific marker for microglial cells, was identified by flow cytometry. Microglial cells were treated with 100 mM methanol.

### 2.7. Cell transfection

Small-interfering RNA targeting KLF6 (si-KLF6) and KLF6 overexpression plasmid (oe-KLF6), miR-124 mimic/inhibitor, and the corresponding NC (GenePharma, Shanghai, China) were transfected into microglial cells based on Lipofectamine™ 2000 (Invitrogen, Thermo Fisher Scientific). After 48 h, the transfection efficiency was determined by reverse transcription quantitative polymerase chain reaction (RT-qPCR).

### 2.8. Co-culture

PC-12 cells were co-cultured with the conditioned medium of microglial cells for 48 h.

### 2.9. Cell Counting Kit-8 (CCK-8)

Cell viability was measured using a CCK-8 kit (Dojindo). PC-12 cells after co-culture with the conditioned medium of microglia treated with different concentrations of methanol (0 mM, 0.1 mM, 1 mM, 10 mM, 100 mM) were added with 10 μL CCK-8 solution, and the absorbance was tested at 450 nm on a microplate reader (Bio-Rad Laboratories, Hercules, CA, USA). Three independent replicates were performed for each group [25].

### 2.9. Flow cytometry

Apoptosis of PC-12 cells was checked by annexin V-fluorescein isothiocyanate (FITC)/propidium iodide (PI) kit (Bestbio Biotechnology Co., Ltd., Shanghai, China). PC-12 cells after detachment with trypsin were re-suspended in 1 × Annexin binding buffer, and 100 μL cell suspension (at a density of 1 × 10^5^) was incubated with 5 μL Annexin V-FITC and 5 μL PI. After incubation, 400 μL 1 × binding buffer was added, and cell apoptosis was determined by Cell-Quest software (BD Biosciences, San Jose, CA, USA) and a flow cytometer (FACSCalibur, BD). Three independent replicates were performed for each group.

To determine the immune types of microglia, cells were incubated with fluorescence-labeled antibodies (CD68, M0876, Dako; CD206, MCA2235, Bio-Rad), fixed with 1% paraformaldehyde and detected using a flow cytometer (FACSCalibur), and Cell-Quest software (BD Biosciences) was used to analyze cell subsets.

### 2.10. RT-qPCR

Total RNA was extracted by TRIzol (Invitrogen) on the grounds of the manufacturer’s protocol. The mRNA and miRNA were subjected to reverse transcription using ReverTra AceqPCR RT kit (Toyobo Co., Osaka, Japan) and TaqMan MicroRNA Reverse Transcription Kit (TaKaRa, Dalian, China), respectively. The qPCR reaction was implemented on an Applied Biosystems machine (Thermo Fisher Scientific, USA) and FastStart Universal SYBR Green Master (Roche, Switzerland). β-actin and U6 were loading controls for mRNA and miRNA, respectively. Data analysis was performed by the 2^−ΔΔCT^ method [26]. Three independent replicates were performed for each group.

### 2.11. Western blot

Cells were lysed with 10 μL/mL Radio-Immunoprecipitation assay Lysis Buffer containing protease inhibitors (Beyotime), centrifuged at 14,000 × g, and quantified by bicinchoninic acid protein assay (Beyotime). Total protein (20 μg) was loaded into a sodium lauryl sulfate polyacrylamide gel and separated. Then, the sample was electroblotted onto a polyvinylidene fluoride membrane (Millipore, Billerica, MA, USA), blocked with 5% skim milk, and incubated with the following primary antibodies: β-actin (A5441, MilliporeSigma), KLF6 (14716-1-AP, Proteintech), Nrf2 (16396-1-AP, Proteintech), NF-κB (14220-1-AP, Proteintech), p-NF-κB (8242, Cell Signaling Technology), HO-1 (10701-1-AP, Proteintech), Bax (50599-2-Ig, Proteintech), Bcl-2 (12789-1-AP, Proteintech), and Ki-67 (27309-1-AP, Proteintech). The membrane was then incubated with the secondary antibody conjugated with horseradish peroxidase (Beyotime), developed by enhanced chemiluminescence kit (Amersham Pharmacia Biotech, Little Chalfont, UK) and imaged by ChemiDoc XRS imaging system. Image J image analysis software was used for data analysis. Three independent replicates were performed for each group.

### 2.12. The luciferase activity assay

The construction of the wild-type (WT) KLF6 3ʹuntranslated region (UTR) reporter plasmid (pmiR-KLF6-wt) and the mutant (MUT) KLF6 3ʹUTR reporter plasmid (pmiR-KLF6-mut) was carried out (GenePharma). The above plasmids with miR-124 mimic and mimic NC were co-transfected into HEK-294 cells. After 48 h, measurement of the luciferase activity was performed using Dual-Luciferase Reporter Assay Kit (Promega, USA) [27]. Three independent replicates were performed for each group.

### 2.13. RNA immunoprecipitation (RIP) assay

The RIP assay was performed with the help of the Magna RIP kit (17–10499-2, Millipore) [28]. Cells were lysed with RIP lysis buffer and incubated with Ago2 antibody or IgG antibody-coupled magnetic beads. After purification, RNA enrichment was detected by RT-qPCR.

### 2.14. Data analysis

GraphPad Prism 9 was used for statistical analysis. Data were shown in the form of mean ± standard deviation. Comparison of differences among multiple groups was implemented by one-way analysis of variance and Tukey multiple comparison test. Comparison of the differences between two groups was done by Student’s *t*-test. *P* < 0.05 was accepted with statistical differences.

## 3. Results

### 3.1. AMP accelerates microglia activation

An AMP rat model was constructed by gavage with methanol. Immunofluorescence staining was applied to observe the specific marker (Iba-1) of microglial cells in the cerebral cortex, showing that AMP increased Iba-1 positive cells in rats (Figure 1(a)). Additionally, flow cytometry identified that AMP increased the number of microglial cells with pro-inflammatory (CD68^+^) and anti-inflammatory (CD206^+^) phenotypes in the cerebral cortex (Figure 1(b)). Subsequently, an examination of inflammatory factors and oxidative stress indices in brain tissue was implemented. As manifested in Figure 1(c,d), AMP elevated TNF-α, IL-1β, IL-6, and MDA while decreased SOD levels. Subsequently, Western blot analysis of inflammatory signaling molecule NF-κB and oxidative stress pathway Nrf2/HO-1 presented that AMP elevated p-NF-κB expression while declined Nrf2/HO-1 expression (Figure 1(e)).

**Figure 1.** AMP accelerates microglial activation. (a,b): Immunofluorescence detection of Iba-1, CD68, and CD206 in AMP rats’ cerebral cortex; (c,d): ELISA test of TNF-α, IL-1β, IL-6, MDA, and SOD in AMP rats’ brain tissue; (e): Western blot examination of p-NF-κB/NF-κB, Nrf2, and HO-1 in AMP rats’ brain tissue; (f): Flow cytometry identification of microglial cell marker Iba-1; (g): Flow cytometry test of CD68^+^ and CD206^+^ microglial cell proportion; (h): RT-qPCR detection of TNF-α, IL-1β, IL-6, MDA, and SOD in microglial cells; (i): Western blot examination of p-NF-κB/NF-κB, Nrf2, and HO-1 in microglial cells. (g–i): after methanol treatment.

Subsequently, the impact of methanol on microglial cells was explored in *in vitro* experiments. Cells were isolated from rat brain tissue, and the isolated cells were identified by flow cytometry to express positive Iba-1 (figure 1(f)). Therewith, microglia phenotypic changes were examined by flow cytometry. As shown in Figure 1(g), methanol treatment promoted the number of CD68^+^ and CD206^+^ microglia. Microglia TNF-α, IL-1β, IL-6, and MDA expression increased after methanol treatment, but SOD expression decreased (Figure 1(h)). Western blot showed that methanol treatment promoted p-NF-κB expression in microglia and inhibited Nrf2/HO-1 expression (Figure 1(i)). To sum up, AMP accelerates microglia activation and stimulates inflammation and oxidative stress in brain tissue.

### 3.2. Elevated miR-124 accelerates M2 polarization

An examination of miR-124 expression after AMP was implemented. As manifested in Figure 2(a), AMP constrained miR-124 expression in brain tissue and microglial cells. Subsequently, miR-124 expression was artificially upregulated in AMP rats and microglial cells (Figure 2(b)). As observed in the cerebral cortex of AMP rats, upregulating miR-124 elevated CD206^+^ cells while reduced CD68^+^ cells (Figure 2(c)), suppressed inflammation and oxidative stress (Figure 2(d, e)), and repressed p-NF-κB protein expression while induced Nrf2/HO-1 protein expression (figure 2(f)). *In vitro* studies further verified the effects of miR-124 (Figure 2(g-i)). In general, elevated miR-124 accelerates M2 polarization.

**Figure 2.** Elevated miR-124 boosts M2 polarization. (a): RT-qPCR test of miR-124; (b): RT-qPCR detection of miR-124 after delivering miR-124 mimic or miR-124 agomir; (c): Immunofluorescence detection of CD68 and CD206 in AMP rats’ cerebral cortex; (d,e): ELISA examination of TNF-α and IL-1β, IL-6, MDA, and SOD; (f): Western blot test of p-NF-κB/NF-κB, Nrf2, and HO-1; (g): flow cytometry detection of CD68^+^ and CD206^+^ microglial cell proportion; (h): RT-qPCR test of TNF-α, IL-1β, IL-6, MDA, and SOD; (i): Western blot test of p-NF-κB/NF-κB, Nrf2, and HO-1. (a,b), in AMP rats’ brain tissue and microglial cells. (d–f), in AMP rats’ brain tissue. (h,i), in microglial cells. (c-i), after elevating miR-124.

### 3.3. MiR-124 targets KLF6

KLF6 is abundant in an imbalance of inflammation and oxidative stress [29]. In this research, AMP elevated KLF6 expression in rat brain tissue and microglial cells, while upregulating miR-124 declined KLF6 expression (Figure 3(a)), given that miR-124 was speculated to target KLF6. MiR-124 and KLF6 had latent binding sites on the website https://starbase.sysu.edu.cn (Figure 3(b)). WT-KLF6 and miR-124 mimic impaired the luciferase activity after co-transfection, while MUT-KLF6 and miR-124 mimic exerted no influence on the luciferase activity (Figure 3(c)). RIP assay found the enrichment of KLF6 and miR-124 after Ago2 treatment (Figure 3(d)). In brief, miR-124 targets KLF6.

**Figure 3.** MiR-124 targets KLF6. (a): Western blot detection of KLF6 in AMP rats’ brain tissue and microglial cells after augmenting miR-124; (b): Bioinformatics website forecast of the latent binding site of miR-124 and KLF6; (c): The luciferase activity assay examination of the targeting of miR-124 with KLF6; (d): RIP experiment test of the enrichment of miR-124 with KLF6 in Ago2 magnetic beads.

### 3.4. Suppression of KLF6 accelerates M2 polarization

The impact of KLF6 on AMP microglia activation was explored. KLF6 in AMP rats and microglial cells were constrained by lentiviral injection and plasmid transfection, respectively (Figure 4(a)). After repressing KLF6, CD206^+^ cells in the cerebral cortex were elevated, while CD68+ cells were decreased (Figure 4(b)), inflammation and oxidative stress were limited (Figure 4(c,d)), p-NF-κB protein expression was reduced, and Nrf2/HO-1 protein expression was elevated (Figure 4(e)). *In vitro* studies also gained consistent results (figure 4(f-h)). In short, suppression of KLF6 accelerates M2 polarization and declines inflammation and oxidative stress.

**Figure 4.** Inhibition of KLF6 accelerates M2 polarization. (a): Western blot detection of KLF6 in AMP rats’ brain tissue and microglial cells after delivering rAVV-sh-KLF6 or si-KLF6; (b): Immunofluorescence examination of CD68 and CD206 in AMP rats’ cerebral cortex; (c,d): ELISA test of TNF-α, IL-1β, IL-6, MDA, and SOD; (e): Western blot detection of p-NF-κB/NF-κB, Nrf2, and HO-1; (f): Flow cytometry detection of CD68+ and CD206+ microglial cell proportion; (g): RT-qPCR examination of TNF-α, IL-1β, IL-6, MDA, and SOD; (h): Western blot test of p-NF-κB/NF-κB, Nrf2, and HO-1. (c–e), in AMP rats’ brain tissue. (g,h), in microglial cells. (b–h), after repressing KLF6.

### 3.5. MiR-124 modulates microglia phenotypic changes via targeting KLF6

MiR-124/KLF6 axis’ action in microglial polarization was explored. MiR-124 inhibitor and si-KLF6 were co-transfected into methanol-treated microglial cells. As presented in Figure 5(a), transfection with miR-124 inhibitor enhanced KLF6 expression, while co-transfection with si-KLF6 prevented this phenomenon. Therewith, microglia phenotypic changes were examined. As presented in Figure 5(b), transfection with miR-124 inhibitor boosted the number of CD68^+^ microglial cells and declined the number of CD206^+^ microglial cells, while co-transfection with si-KLF6 prevented M1 polarization. Subsequently, inflammatory factors and oxidation indices were inspected. As manifested in Figure 5(c), transfection of miR-124 inhibitor promoted inflammation and oxidative stress, but co-transfection with si-KLF6 turned around the effect of miR-124 inhibitor. Western blot found that transfection with miR-124 inhibitor accelerated p-NF-κB expression in microglial cells and constrained Nrf2/HO-1 expression, while co-transfection with si-KLF6 prevented this phenomenon (Figure 5(d)). In brief, miR-124 modulates microglia phenotypic changes via targeting KLF6.

**Figure 5.** MiR-124 modulates microglial phenotypic changes via targeting KLF6. (a): Western blot detection of KLF6; (b): Flow cytometry test of CD68+ and CD206+ microglial cell proportion; (c): RT-qPCR examination of TNF-α, IL-1β, IL-6, MDA, and SOD; (d): Western blot detection of p-NF-κB/NF-κB, Nrf2, and HO-1. (a–d), after co-transfecting miR-124 inhibitor with si-KLF6. (a,c,d), in microglial cells.

### 3.6. MiR-124/KLF6 axis influences neuronal viability and apoptosis via mediating microglial cell polarization

Whether the regulation of microglial polarization by the miR-124/KLF6 axis affects neuronal apoptosis was explored. The conditioned medium of microglial cells was co-cultured with neurons. An examination of neuronal cell viability (Figure 6(a-d)) elucidated that the conditioned medium of microglial cells treated with 100 mM methanol had the extremely high cytotoxicity to neurons. As observed, the conditioned medium reduced neuronal viability and protein expression of Ki-67 and Bcl-2 and promoted neuronal apoptosis and Bax expression. Knockdown of miR-124 further promoted neuronal damage caused by the conditioned medium, but this phenomenon was reversed by knockdown of KLF6. These results suggest that miR-124/KLF6 affects neuronal viability and apoptosis by regulating microglial polarization.

**Figure 6.** The miR-124/KLF6 axis impacts neuronal activity and apoptosis via modulating microglial cell polarization. (a): CCK-8 detection of the impacts of co-culture with CM of microglial cells treated with different concentrations of methanol (0, 0.1, 1, 10, 10, 100 mM) on cell viability; (b): CCK-8 test neurons’ cell viability; (c): Flow cytometry examination of neurons’ apoptosis rate; (d): Western blot detection of Ki-67, Bax, and Bcl-2 in neurons. (b–d), co-cultured with CM.

## 4. Discussion

AMP is available to lead to severe damage to the central nervous system (CNS) [30]. Momentous progress has been made in AMP treatment, but the mortality rate is still increasing. Studies have elucidated the action of neuroinflammation in AMP-stimulated toxic brain injury [31], and numerous evidences have illuminated that miRNA is implicated in mediating all aspects of neuronal dysfunction and neuroinflammation [32]. For instance, miR-152 mitigates neuroinflammation in cerebral hemorrhage [33]. In this study, miR-124 modulated microglial polarization via targeting KLF6, thereby influencing neuroinflammation in AMP. The results clarified that miR-124 might become a novel therapeutic target for AMP-stimulated neuroinflammation.

As reported, microglia are CNS resident cells involved in immune surveillance and maintenance of intercellular homeostasis [34]. Neuroinflammation is mediated by microglia, which modulate the progression of neuroinflammation by transitioning to a distinct phenotype [9]. In multiple neurological diseases, microglia transition from M1 to M2 phenotype heralds disease improvement and functional recovery [35]. For a long time, Iba-1, CD86, and CD206 have been considered biomarkers of microglial activation; Increased Iba-1 expression indicates microglial activation, while CD86 and CD206 serve as M1 and M2 status markers, respectively [36]. In this research, Iba-1 in AMP rats’ cerebral cortex was augmented, and the number of microglial cells of pro-inflammatory (CD68^+^) and anti-inflammatory (CD206^+^) phenotypes was elevated as well. Additionally, inflammatory indicators in AMP rats’ brain tissue were augmented. These results manifested that AMP accelerated microglial activation and stimulated neuroinflammation.

Mitochondrial dysfunction is available to stimulate ROS in cells, leading to oxidative stress [37] and oxidative stress is associated with microglial activation [38]. Microglial activation may increase pro-inflammatory cytokine production, which in turn promotes ROS to accelerate oxidative stress, and increased ROS production increases inflammatory cytokine production and enhances microglial activation by stimulating NF-κB [39]. As detected, AMP promoted microglia activation; therefore, it was speculated that AMP also induces oxidative stress. MDA and SOD reflect the state of oxidative stress, while Nrf2, a redox-sensing transcription factor, is available to drive adaptive cellular defenses in response to oxidative stress [40]. In the research, AMP led to increased levels of MDA and phosphorylated NF-κB in brain tissue and decreased levels of SOD and Nrf2/HO-1, while overexpression of miR-22-3p or knockdown of KLF6 alleviated the effect of AMP and maintained oxidation and antioxidant balance, which will contribute to the transformation of microglia to an anti-inflammatory type.

miRNA mediates microglial activation by modulating the NF-κB pathway. For instance, miR-183 controls the microglial activation in rats with cerebral ischemia-reperfusion injury via constraining the NF-κB pathway [41]. MiR-873a-5p mitigates microglial cell-mediated neuroinflammation and ameliorates neurological deficits after traumatic brain injury via restraining the NF-κB pathway [42]. In this research, miR-124 was down-regulated in AMP rat brain tissue and microglia, indicating that miR-124 is a stress-responsive miRNA. Furthermore, it was tested that miR-124 overexpression declined NF-κB phosphorylation in the cerebral cortex, inflammation, and the number of CD68^+^ microglial cells and accelerated Nrf2/HO-1 and the number of CD206^+^ microglial cells. These data elucidated that in AMP rats, miR-124 influenced inflammatory factors via modulating the NF-κB pathway, thereby mediating M2 polarization. Recently, several studies have demonstrated circulating miRNAs as potential biomarkers of alcohol-induced neuroinflammation [43]. Although this study has not yet examined the expression of miR-124 in the serum of AMP patients or animals, it is worth confirming in follow-up studies to develop novel clinical diagnostic markers for AMP.

KLF6, a nuclear transcription regulator, mediates various cellular processes [44]. KLF6 is a co-activator of NF-κB, and overexpression of KLF6 enhances TNF-α and IL-1β-induced NF-κB activation and transcription of downstream genes, whereas KLF6 knockdown reverses this phenomenon [45]. In this study, KLF6 was elevated in AMP rats’ brain tissue and microglial cells, and KLF6 knockdown has the same result as upregulation of miR-124. However, a foregoing study has elaborated that miR-124 might target KLF6 mRNA [46]. Consequently, KLF6 was speculated to be a downstream target gene of miR-124. Further experiments testified that miR-124 modulated microglial phenotypic changes via targeting KLF6. Additionally, researchers have elaborated that continued overactivation or loss of control of microglia can induce the release of various cytotoxic factors and aggravate neuronal damage [47]. Consequently, miR-124/KLF6 axis’ impacts on microglial polarization in neurons were explored, ultimately proving that knockdown of miR-124 promoted neuronal damage by AMP, but this phenomenon was reversed by knockdown of Ki-67.

## 5. Conclusion

In brief, our findings are the first to identify a novel regulatory mechanism of neuroinflammation in AMP rats, demonstrating that miR-124 regulates neuroinflammation by targeting KLF6 to modulate microglial polarization in the cerebral cortex of rats with AMP by modulating neuronal viability and apoptosis. This will aid in the development of future approaches to modulate microglial activation during neuroinflammatory and neurodegenerative diseases. However, the present study has not demonstrated the clinical role of the miR-124/KLF6 axis in AMP. The clinical effect of MiR-124/KLF6 axis needs to be confirmed in follow-up studies. Furthermore, the whole brain homogenate was examined in this study, and the specific role of miR-124/KLF6 is unclear. Does it have effects on epidermal cells or immune cells? This needs to be explored in follow-up research.

## Supplementary Material

Supplemental Material
